The article "On the Design of Secured and Reliable Dynamic Access Control Scheme of Patient E-Healthcare Records in Cloud Environment" was retracted in 2023. Reasons: signs of a paper mill; suspected computer-generated content; unreliable results or conclusions; concerns about the data.

# On the Design of Secured and Reliable Dynamic Access Control Scheme of Patient E-Healthcare Records in Cloud Environment

**DOI:** 10.1155/2022/3804553

**Published:** 2022-08-18

**Authors:** Kirtirajsinh Zala, Hiren Kumar Thakkar, Rajendrasinh Jadeja, Neel H. Dholakia, Ketan Kotecha, Deepak Kumar Jain, Madhu Shukla

**Affiliations:** ^1^Department of Computer Engineering, Marwadi University, Rajkot 360006, Gujarat, India; ^2^Department of Computer Science and Engineering, School of Technology, Pandit Deendayal Energy University, Gandhinagar 382007, Gujarat, India; ^3^Faculty of Technology, Marwadi University, Rajkot 360006, Gujarat, India; ^4^Symbiosis Centre for Applied Artificial Intelligence, Symbiosis International (Deemed) University, Pune, India; ^5^Key Laboratory of Intelligent Air-Ground Cooperative Control for Universities in Chongqing, College of Automation, Chongqing University of Posts and Telecommunications, Chongqing, China

## Abstract

Traditional healthcare services have changed into modern ones in which doctors can diagnose patients from a distance. All stakeholders, including patients, ward boy, life insurance agents, physicians, and others, have easy access to patients' medical records due to cloud computing. The cloud's services are very cost-effective and scalable, and provide various mobile access options for a patient's electronic health records (EHRs). EHR privacy and security are critical concerns despite the many benefits of the cloud. Patient health information is extremely sensitive and important, and sending it over an unencrypted wireless media raises a number of security hazards. This study suggests an innovative and secure access system for cloud-based electronic healthcare services storing patient health records in a third-party cloud service provider. The research considers the remote healthcare requirements for maintaining patient information integrity, confidentiality, and security. There will be fewer attacks on e-healthcare records now that stakeholders will have a safe interface and data on the cloud will not be accessible to them. End-to-end encryption is ensured by using multiple keys generated by the key conclusion function (KCF), and access to cloud services is granted based on a person's identity and the relationship between the parties involved, which protects their personal information that is the methodology used in the proposed scheme. The proposed scheme is best suited for cloud-based e-healthcare services because of its simplicity and robustness. Using different Amazon EC2 hosting options, we examine how well our cloud-based web application service works when the number of requests linearly increases. The performance of our web application service that runs in the cloud is based on how many requests it can handle per second while keeping its response time constant. The proposed secure access scheme for cloud-based web applications was compared to the Ethereum blockchain platform, which uses internet of things (IoT) devices in terms of execution time, throughput, and latency.

The article "On the Design of Secured and Reliable Dynamic Access Control Scheme of Patient E-Healthcare Records in Cloud Environment" was retracted in 2023. Reasons: signs of a paper mill; suspected computer-generated content; unreliable results or conclusions; concerns about the data.

## 1. Introduction

In the recent past, data volumes are exponentially increased each passing day due to affordable and easy access to internet-enabled connected devices [1, 2]. The healthcare systems are under constant strain to deal with a high volume of healthcare data with the expectation to predict the results in a reasonable time duration. Systems and algorithms are developed to deal with the high velocity of the healthcare data for efficient prediction. However, most of such systems are subject to data security risk and face attacks such as denial of service (Dos), snooping, and traffic analysis [3]. In addition, the recent coronavirus pandemic has forced the hospitals to run at overcapacity making it difficult to keep patient records secure. The conventional method of manual handwritten paper-based information storage is not viable and makes it difficult to efficiently retrieve the data. Moreover, traditional methods make it challenging to find a patient's individual medical and data that are subject to be lost or destroyed [4]. Using blockchain and Interplanetary File System (IPFS), the author [5] proposes an architecture that aims to offer quicker retrieval and consistent personal health record availability. The findings demonstrate that an ideal node is chosen among all potential adjacent nodes in each iteration.

The internet of things (IoT) technology enables the storage of health records in digital format [6, 7]. Because e-healthcare security includes the patient's confidential health information, it is more essential to be in a secured form. To carry out attacks, attackers can take advantage of the vulnerabilities in open wireless channels [8–11]. These attacks have the potential to harm the e-healthcare system in various ways. An example of this would be a patient who has been treated and then sent home from a hospital in a place other than his own. The patient later becomes ill and is hospitalized nearby, but it does not have all of the data or the records from his previous hospitalization. Due to a lack of information, his therapy may be delayed or fatal. However, if the patient's data are already stored on cloud-connected devices, retrieving the patient's data takes only seconds, allowing the new hospital personnel to begin treatment earliest possible [12].

The article "On the Design of Secured and Reliable Dynamic Access Control Scheme of Patient E-Healthcare Records in Cloud Environment" was retracted in 2023. Reasons: signs of a paper mill; suspected computer-generated content; unreliable results or conclusions; concerns about the data.

Using high-security cryptography techniques, the healthcare department can keep encrypted data in the cloud, limiting access to only those who have been granted permission. The cloud comprises servers that run various software and databases and can be accessed via the internet. Cloud servers can be found worldwide to store and access data from any place, anywhere. Because of cloud computing, the healthcare departments and insurance companies do not need to make use of any physical servers or any software programs [13]. The capacity to quickly and securely transfer massive volumes of data, such as patient medical records, is one of the many advantages of cloud computing [14]. Healthcare providers should use digital solutions in hospitals to ensure that their infrastructure is well managed and that they have adequate opportunities to engage themselves with IT service providers [15, 16]. Cost-effectiveness, collaborative resource sharing, scalability, and agility enhancement are some of the other advantages of mobile and cloud computing [17].

Electronic health data (EHD), personal health record (PHR), and electronic medical record (EMR) are all types of digital medical records [18]. Healthcare professionals keep EMR and EHR, whereas the patients or their relatives own PHR. Man-in-the-middle attack, denial of service (DOS), eavesdropping, and so on are all threats to wireless communication among physicians and patients, and between the cloud and the systems.

Healthcare providers and patients can benefit from the cloud's ability to store, process, and update information without spending a lot of money and its ability to make things more efficient and of better quality. Since this information is stored on more than one server, it can be easily accessed from many different places. E-health systems guarantee on-demand, quick, and consistent access to health records, and fewer medical errors and higher-quality treatment. But they also leave patient privacy open to misuse of EHR data and improper authorization. So, security and privacy are very important when multiple people share or look at patient data.  Figure 1 gives an overview of the architecture of e-health.

Although cloud services offer enormous benefits, they still face numerous security risks. The cloud service provider, for example, has a vast amount of data that users do not know about [19]. A lack of transparency makes it impossible to know how data are handled and where. Because of this, it is harder to have faith in the service provider, and data loss may result.  Figure 1 shows the vulnerability of untrusted servers to assaults from both internal and external adversaries because they lack privacy-preserving safeguards.

The article "On the Design of Secured and Reliable Dynamic Access Control Scheme of Patient E-Healthcare Records in Cloud Environment" was retracted in 2023. Reasons: signs of a paper mill; suspected computer-generated content; unreliable results or conclusions; concerns about the data.

The CP-ABE systems with multiple authorities and threshold secret sharing (*t*, *n*) can be integrated; this research [20] presents an improved security and performance for public cloud storage by addressing the single-point bottleneck problem, which enhances both security and performance. Using an auditing technique, a solitary bottleneck issue for the most existent CP-ABE systems can be alleviated, according to the author [21]. E-health cannot benefit from these advanced access control schemes [20, 21] despite the fact that the central authority and many attribute authorities cannot ensure protection from insider attacks, even though they are advanced access control schemes with excellent security measures. Water-based CP-ABE (cyphertext-policy attribute-based encryption) system deniable on attribute-based encryption (ABE) technique is a particular encryption approach that allows cloud storage providers to build fake user identities using preserved cyphertext in order to safeguard data from external attackers [22].

By encrypting data belonging to many patients who share the same access policy mentioned by [23], the author's system offers multiprivileged access control for personal health records (PHRs). For disease prediction, author [24] uses the single-layer perceptron learning algorithm. Using encrypted prediction models developed by this model, the cloud leverages encrypted symptom data supplied by patients to diagnose their illness without jeopardizing patient privacy. Health records cannot benefit from these procedures because of their high level of data privacy and computational complexity and scalability concerns [23, 24]. A CP-ABE with the disguised access control mechanism policy and permitted access control was proposed in another study, [25].

A new identity-based encryption (IBE) method based on revocable storage presented by the author [26] protects cyphertext in both the forward and backward directions. There is currently no dynamic user management among the most secure provenance cloud storage systems, which results in considerable performance overhead and poor access control. An attribute-based, provenance-assured cloud storage system is presented in this paper [27], which offers an answer to the issue. As efficient as ABE schemes are, it is still not possible to implement them on EHRs. This is despite the fact that ABE schemes provide perfectly alright, well-formed access to health records [25, 27]. There are several reasons for this, including high computing costs, the difficulty of managing keys, and the inability to effectively administer access control regulations [22]. A policy that offers approved access control with a constant key length increases as the number of attributes in the access structure increases [25].

The article "On the Design of Secured and Reliable Dynamic Access Control Scheme of Patient E-Healthcare Records in Cloud Environment" was retracted in 2023. Reasons: signs of a paper mill; suspected computer-generated content; unreliable results or conclusions; concerns about the data.

The e-healthcare technology should also protect patient's data, even if the healthcare department argues that personnel are responsible for doing so. Our study suggests a system in which only authorized personnel have access to patient information. The doctor has read and wrote access to the data, whereas others can only read it but not edit it. To guarantee the protection of sensitive data from beginning to end, the suggested technique outlines how an administrator generates subkeys with help of the master key. Confidentiality, authenticity, and protection from known critical attacks were all included in our study of healthcare system security [28, 29].

### 1.1. Motivation and Contribution

There are not enough privacy protection systems in place to guarantee complete safety in the cloud for e-health data. Health records kept on cloud servers face the greatest risk from insider assaults, such as those by database administrators or key managers, rather than outsiders as it is contrary to popular opinion. Furthermore, cloud access could expose potentially sensitive information to malicious users if not secured. Risks to patient's lives increase as a result of its medical usage. The malicious user may also use the information to harm the hospital's reputation. Future solutions to these cyberattacks and criminal individuals may include the adoption of secure access control technologies. However, due to asset user devices and insecure wireless channels, it is challenging to build such protocols. As a result, lightweight security mechanisms with excessive reliability should be developed to protect sensitive patient data over the third-party cloud service provider.

- We created a single cloud-based web application used to store and provide secure access to e-health records from anywhere. The web application is hosted on the AWS (Amazon Web Services) cloud platform by launching multiple instances. We also investigated the performance of our web application in terms of specific requests per second. Performance is evaluated by looking at resource provisioning, CPU utilization, throughput, and response time.
- We compared the performance evolution of a secure access scheme for a cloud-based web application for patient health records with the Ethereum blockchain platform using IoT devices.
- We propose a bold and secure method of entry for e-healthcare services in the cloud-based scheme.
- In accordance with the recommended security protocols, only legitimate users can use cloud services, which confirm the user's identification in cloud-based e-health application (patient, doctor, and ward boy).
- The proposed protocol protects networks from message modification, replay, and man-in-the-middle attacks while ensuring data confidentiality, message freshness, and other security features.

The article "On the Design of Secured and Reliable Dynamic Access Control Scheme of Patient E-Healthcare Records in Cloud Environment" was retracted in 2023. Reasons: signs of a paper mill; suspected computer-generated content; unreliable results or conclusions; concerns about the data.

The rest of this paper is organized as follows.  Section 2 discusses the literature review, Section 3 describes the system design and adversary prototype, Section 4 explains the proposed scheme for secure access, Section 5 presents the experimental setup with results and discussion, Section 6 discusses experimental design, and Section 7 ends with the conclusion.

## 2. Literature Review

According to a study [30], a new web-based solution that allows doctors, ward boys, and pharmacists to access patients' medical records has been developed. It stores the patient's information on the local cloud. The data can be accessed and updated from a distance. To collaborate on treatments, records must be provided to other doctors. The disadvantage in the method is it prevents patients from accessing their medical records.

The researchers of [31] proposed a healthcare framework based on the cloud for effective collaboration among caregivers and the healthcare providers, which might fully change hospital's handwritten record systems. The records can be accessed by healthcare providers and patients from any location utilizing the system. The authorization management service, part of the framework, could only be accessed by a genuine healthcare practitioner or patient. In contrast to patients, healthcare professionals are allowed to write, read, and alter the data. There are two portions to a patient's health record; one is locally stored in a healthcare facility, while another is stored on a cloud database server. The biggest issue with this approach is that the cloud server stores all data when a hospital or healthcare facility does not have a local EHR system.

In paper [32], experts examined, studied, and evaluated several papers and found that several issues need to be addressed to preserve e-healthcare records (EHR). EHR security, EHR cloud architecture, and EHR privacy are only a few. The authors also state that there are still many studies to be performed in the field of EHR security. Author [33] proposes a solution to the problem of managing user access control to a complex universe of user data while maintaining confidentiality while storing medical records in the cloud. Author [34] described an authentication method for an EHR system with a hybrid cloud structure, allowing us to handle different types of users with varying access privileges.

The authors [35] propose a simple and effective method for securing healthcare institution collaboration. They present secure multiparty computation (SMC) methods to assure compliance with data protection regulations. When outsourcing computations to the public cloud, the authors employ the Paillier scheme to safeguard medical data from unauthorized access. Another advantage of this technique is its ability to execute arithmetic operations on encrypted data without access to the original data. Using Shamir's secret sharing, the author proposes a novel cloud storage system for EHRs that ensures data privacy in its entirety. In this system, a healthcare facility divides an EHR into multiple segments, which are then distributed to numerous cloud servers. When retrieving EHRs, the healthcare facility extracts segments from partial cloud servers and reconstructs EHRs [36].

The article "On the Design of Secured and Reliable Dynamic Access Control Scheme of Patient E-Healthcare Records in Cloud Environment" was retracted in 2023. Reasons: signs of a paper mill; suspected computer-generated content; unreliable results or conclusions; concerns about the data.

The suggested method listed in paper [37] is based on the FHE (fully homomorphic encryption) algorithm with key delegation to ensure data privacy, authentication, integrity, and availability in a hierarchical structure with multiple levels. This will give the healthcare provider the freedom to use or not use any access rule in any order, which is especially important in a medical research setting. Still, there is more work to be done to make FHE really useful. Flow-enabled distributed mobility anchoring (FDMA) was proposed by the author to reduce signaling overhead cost (SOC) and packet tunneling cost (PTC) [38].

The researcher in paper [39] presents the experimental investigation of cryptographic algorithms to classify encryption algorithm types such as symmetric and asymmetric. It provides a comprehensive analysis of advanced encryption standards (AES), data encryption standards (DES), 3DES, RSA, and Blowfish in terms of timing complexity, file size, encryption, and decryption performance. The speed of encryption and decryption of the selected encryption algorithms has been evaluated utilizing a simulation-based methodology. The research [40] proposes using the distributed fog computing architecture that uses the elliptic curve Diffie–Hellman ephemeral (ECDHE) key exchange algorithm with the preshared key (PSK) as an authentication method that is both lightweight and safe. As an alternative to the static PSK technique, the ephemeral preshared key used by the ECDHE-PSK authentication system provides perfect forward secrecy (PFS). Literature [41] provides a lightweight, reliable encryption scheme for healthcare image encryption.

The purpose of paper [42] is to discuss data security and authentication in the healthcare industry. Author [43] has proposed a blockchain-based, public-key cryptography-based secure framework. The authors of [43] suggest a model in which medical pictures from the Digital Imaging and Communications in Medicine (DICOM) standard, which contains data on disease and may be applied in real time to the healthcare system, are shared. Due to the blockchain-based decentralized storage model, the framework keeps the immutability, privacy, and availability of information. They also discussed how peers inside the blockchain network could access information via consensus, which they explained in detail. To solve the problem of scalability, the author [44] suggests an improved version of the Bell–LaPadula model and divides peers and transactions into groups with different levels of clearance and security. Due to the clearance level, the peers do not have to keep track of every transaction made. Using smart contracts, author set up dynamic access control policies in the network to keep data safe. Author uses a blockchain-based healthcare network to test their model [44].

The article "On the Design of Secured and Reliable Dynamic Access Control Scheme of Patient E-Healthcare Records in Cloud Environment" was retracted in 2023. Reasons: signs of a paper mill; suspected computer-generated content; unreliable results or conclusions; concerns about the data.

Today, this large amount of medical data made by IoMT (internet of medical things) is kept in a centralized storage system. However, centralizing all of a patient's private information raises questions about security and privacy. To deal with these problems, author suggests a consortium blockchain network that can handle smart contracts. In the initial stage of patient and medical device authentication, the author built an integrated interplanetary file system cluster node that is an interplanetary file system using smart contracts. In order to safely transfer device-generated data throughout the consortium blockchain, it is proposed that the same cluster layer has been used as a distributed data storage layer [45].

After the study of various comparative literature review of cryptographic and noncryptographic methods, decentralized EHR of patient for legitimate users with centralized management of patient data security is one of the most challenging problems when using cloud systems. It is one of the main reasons why many organizations in e-healthcare avoid using cloud services. The issue is how cloud systems for integrating decentralized information systems must be constructed in terms of technology and organization so that cloud user privacy laws may be guaranteed. Our paper proposes a secure scheme implemented in a cloud-based e-health application in which only authorized personnel can access patient data. Those outside of the doctor's office can only view the data, but they are unable to change or add to the information. The proposed scheme implemented in cloud-based e-health application is designed for decentralized EHR with centralized management. Moreover, in the industrial IoT, there is a growing demand for a privacy-preserving secured framework. In [46], a deep blockchain-based trustworthy privacy-preserving secured framework in the industrial internet of things systems is proposed.

The article "On the Design of Secured and Reliable Dynamic Access Control Scheme of Patient E-Healthcare Records in Cloud Environment" was retracted in 2023. Reasons: signs of a paper mill; suspected computer-generated content; unreliable results or conclusions; concerns about the data.

Patient EHRs are decentralized in terms of providing selected rights to third parties (doctors, ward boys, relatives, and hospitals) with access to critical resources (information, applications, EHR, and reports) to enable more effective operations in application. The “Storage Cloud” cloud computing technology is suitable for the technological implementation because it facilitates the simple incorporation of user data storage into the system. Data administration and authoritative authority are delegated to a centralized service provider that does not store user data. The user acquires a greater degree of responsibility and authority as a result of the breakdown of trust. A guarantee of data availability is essential for the provision of high-quality services. Applications containing EHR are run in a decentralized manner but are centrally managed.

### 2.1. Comparative Analysis of Proposed Scheme

Table 1 provides a clear comparison of the security features of the existing and new protocols. The suggested approach achieves all of the significant security features, for example, secrecy, integrity, authorization, anonymity, and authentication, as shown in the first row of Table 1. On the other hand, traditional approaches cannot achieve all of them, as evidenced by all except the first row of the table. The failure of any standard system to accomplish all basic security features indicates potential weaknesses and high attack possibilities.

Table 2 compares and contrasts the different protocols on e-healthcare security. Table 2 details that many risks attackers can use to launch cyberattacks against different medical devices. Table 2 includes the level of complexity required to successfully hack into medical devices and the level of awareness that stakeholders must have in order to successfully hack into them. The strategies in some of the research paper presented here in literature review do not provide perfect security regarding authenticity, anonymity of one's identity, communication integrity, and secrecy. Because traditional schemes lack these security features, they are unsuitable for sensitive e-healthcare applications. Adversaries can invade and obtain unlawful resources due to flaws in the structure of existing methods. Furthermore, traditional systems have high processing and transmission costs, depriving tiny, intelligent nodes of valuable resources. E-healthcare apps require a sophisticated, authenticated vital agreement method to safeguard the network against unauthorized misuse.

The article "On the Design of Secured and Reliable Dynamic Access Control Scheme of Patient E-Healthcare Records in Cloud Environment" was retracted in 2023. Reasons: signs of a paper mill; suspected computer-generated content; unreliable results or conclusions; concerns about the data.

The proposed scheme's advantages and disadvantages are as follows:

1. Resilient against repeated attacks.
2. Protected against “man-in-the-middle” (MITM) attacks.
3. Protected from attacks that modify the data.
4. The proposed method protects the confidentiality of the data.
5. The proposed scheme demonstrates authorization from legally responsible different stakeholders

However, the disadvantage is when used with low-power wide area networks, the proposed scheme does not result in cost saving when using a local database. This is the possibility for the scheme's future development to turn into a more affordable low-power wide area network solution. As a result of the investigation, the proposed system is seen to be superior to the traditional schemes.

## 3. System Design and Adversary Prototype

### 3.1. System Design

The admin, gateway (*G*_*T*_), patient, ward boy, and doctor relationships are described in the system design.  Figure 2 illustrates how stakeholders could access cloud-based health records via gateway.

### 3.2. Central Administrator

A hospital's IT director serves as the central administrator and registers the facility in the cloud. The administrator securely interacts with the cloud by way of the gateway using the public key of that cloud. The cloud calculates the hospital's master key and returns it to the administrator upon registration. Subsequently, the administrator uses KCF (key conclusion function) to produce numerous subkeys from the master key. The administrator also registers the doctor, ward boy, and patient's devices offline and assigns subkeys to them.

### 3.3. Doctor

A doctor is responsible for treating the patients who have been assigned to him. The patient's data should only be accessible to the doctor who is related to the patient. Comparing the cloud-based patient ID here to the patient ID provided by the doctor is how it is accomplished, and if a match is found, the request is approved; otherwise, the request is denied. Access to editing/writing of a patients' medical record is available to the doctor based on his treatment. The doctor uses encryption, hashing, and subkeying to save all of the patient's data on the cloud. The information can only be read by those who have been granted access. The doctor provides the administrator with two unique identifiers, *ID*_*UG*_ and *ID*_*UH*_. They are kept in the cloud by the administrator. Cloud generates a one-of-a-kind *DR*_*I*  *D*_ number. To connect securely with the gateway, a doctor uses the confidential subkey issued by the admin.

### 3.4. Patient

The hospitalized person for a diagnosis or examination is referred to as the patient. A specific ward boy and doctor are allocated to care for patient in the hospital based on patient diagnosis. The patient additionally gives the administrator two unique identifiers supplied by the government (*ID*_*UG*_) and by the hospital (*ID*_*UH*_). The administrator gets both identifiers and keeps them in the cloud. The administrator receives the unique patient identifier (*PT*_*I*  *D*_) from the cloud. A patient must have the administrator's secret subkey to safely communicate with the gateway. We can assume that the devices of the stakeholders are resource constrained.

The article "On the Design of Secured and Reliable Dynamic Access Control Scheme of Patient E-Healthcare Records in Cloud Environment" was retracted in 2023. Reasons: signs of a paper mill; suspected computer-generated content; unreliable results or conclusions; concerns about the data.

### 3.5. Ward Boy

After the doctor has left, the patient is cared for by a ward boy. Ward boy gets the data from the cloud through a gateway using his subkey *K*_*S*_. The ward boy supplies her government-issued unique identity number (*ID*_*UG*_) and the hospital's address when registering offline (*ID*_*UH*_). The ward boy receives the administrator's secret subkey *K*_*S*_ and the cloud's *NS*_*I*  *D*_ (ward boy ID). A ward boy can only see the information about the patients who have been allocated to him through the healthcare department. The patient's EHR does not allow a ward boy to update or write information in it; thus, he is only able to view the data rather than alter it. Ward boy uses his private subkey issued by the administrator to securely interact with gateway, and it is considered that user's devices have limited resources.

### 3.6. Relative

Relative is role which patient from its dashboard can assign. Patient can give specific access rights of its e-healthcare records stored on cloud environment from its dashboard. If patients are in critical condition or cannot share their health records from a third-party cloud, relative can access their health records and consult a doctor.

### 3.7. Gateway

When a user wants to access the cloud, they can do so through a gateway. The gateway is resource-unrestricted in the present system paradigm, centered on the hospital's applications. The gateway creates a secure interface for the doctor, ward boy, and patient that too view their cloud records after receiving their complete security credentials from the administration. The gateway obtains the master key *K*_*M*_, and subkeys *K*_*S*_ and *HP*_*I* *D*_ through the administrator during offline registration. The doctor, ward boy, and patient communicate with the gateway via distinct subkeys while the gateway and cloud communicate via the master key (*K*_*M*_); the gateway uses encryption to protect their communications.

### 3.8. Adversary Prototype

To disrupt normal network and service operations, hostile nodes are employed. This new protocol's ability to withstand hostile operations was evaluated using the Dolev–Yao adversary model (DY model). Messages transmitted between a gateway, a user, and the cloud can be intercepted by an adversary, according to the DY model. A hacker can intercept and replay user authentication messages en route to the cloud to illegally access cloud services. Intercepted communications may reveal secret credentials that the adversary can use for attacks like man-in-the-middle or known key emulation. An opponent can also launch a DoS attack by repeatedly bombarding the cloud.

The article "On the Design of Secured and Reliable Dynamic Access Control Scheme of Patient E-Healthcare Records in Cloud Environment" was retracted in 2023. Reasons: signs of a paper mill; suspected computer-generated content; unreliable results or conclusions; concerns about the data.

## 4. Proposed Scheme for Secure Access

For any hospital, keeping track of patients and their data is a major concern for the staff; therefore, they have to multitask at all times. The solution we provided was for medical records to be stored in the cloud, saving hospital staff time and effort by eliminating the need to manually enter data. We consider the following assumptions in order to run the proposed methodology:

- Although the user's device has limited computational and storage resources, the cloud and gateway are well-known entities with enormous compute and storage capacities.
- The user device, cloud, and the gateway can perform cryptographic functions.
- Data can only be accessed by a user who has been authenticated in the cloud.

The key conclusion function (KCF) is a cryptographic function for generating more than one secret keys using a master key (KCF). KCF can be used to stretch keys to make them longer or to get the keys in the desired format. The key derivation function, in this case, KCF, serves as good example of pseudorandom function. In this case, the derived key is *D*_*K*_ and the key conclusion function is KCF. The suggested approach comprises four stages: registration for hospital, data retrieval, data storage, and offline registration.

### 4.1. Registration for Hospital

The notations used all over the paper are listed in Table 3.  Figure 3 depicts the administration's cloud registration process with the hospital via gateway. The nonce (*N*_CC1_) is generated by administrator, who concatenates these values *RR*_*N*_‖*RP*_*N*_‖*HP*_ID_‖*N*_CC1_ for formation of *ε*. The message *ε* is encrypted with *CK*_*PU*_ forming *υ*, and the resulting message (*M*_01_) is forwarded to the gateway. The message *υ* is received by the gateway, by which the nonce is generated *N*_CC2_, which gets encrypted using *CK*_*PU*_ to create *ι*. The encrypted message gets in series with *υ* to *α*, and subsequently, the generated message *M*_02_ is delivered to the cloud. The message received gets decrypted with *CK*_*PR*_ for computing *β*, and then, *N*_CC2_ is generated. The cloud checks the nonce *N*_CC2_'s freshness. The procedure is continued if *N*_CC2_ is fresh; otherwise, it is aborted. To compute F, the cloud uses *CK*_*PR*_ to decrypt the message *υ*. Cloud also checks the nonce *N*_CC1_ for freshness; if it is, the process is continued; otherwise, it is cancelled. The cloud checks *RR*_*N*_‖*RP*_*N*_‖*HP*_*I*  *D*_ and aborts the procedure if they are not found to be true. The master key *K*_*M*_ and nonce *N*_CC3_ and *N*_CC4_ are now generated by the cloud. To compute *G*, all values are concatenated *HP*_*I*  *D*_‖*K*_*M*_‖*N*_CC3_. By concatenating and hashing, *H*_*S*_ (*RR*_*N*_‖*RP*_*N*_‖*HP*_*I*  *D*_‖*N*_CC1_), cloud additionally computes KY_AT_ at this point. A key, KY_AT_, is used to encrypt the computed value *G*. *KY*_*GT*_ = *H*_*S*_ is obtained by using hash function (*N*_CC2_). To construct L, the gained key, KY_GT_, is used for the encryption of the nonce *N*_CC4_. The messages L and *K* are concatenated and then stored in *M*. The gateway receives the message *M*. The KY_GT_ gets calculated by the gateway using the hash of *N*_CC2_. KY_GT_ is used to decrypt the message *L*, resulting in *R*. The purity of *N*_CC4_ is tested, and if it is found to be true, the process is restarted; otherwise, it is stopped. The value *K* is sent to the admin as a message *M*_04_ by the gateway. To construct KY_AT_, administrator evaluates the hash value of *DR*_*I*  *D*_‖*PT*_*I*  *D*_‖*D*_*RQ*_‖*N*_*CC*4_. To create *Y*, the received message *K* is decrypted with KY_AT_. The purity of nonce *N*_CC3_ is tested at this point, and if it is determined to be pure, the procedure is resumed. Finally, the administrator can successfully obtain the master key (*K*_*M*_). This master key is a secure communication between the gateway and the cloud through the secret key.

The article "On the Design of Secured and Reliable Dynamic Access Control Scheme of Patient E-Healthcare Records in Cloud Environment" was retracted in 2023. Reasons: signs of a paper mill; suspected computer-generated content; unreliable results or conclusions; concerns about the data.

### 4.2. Offline Registration

Registration method of offline device registration is shown in Figure 4. The administrator keeps track of each stakeholder's unique identifying information, such as *ID*_*UG*_ and *ID*_*UH*_. As identifying data, the gateway provides the administrator with the MAC address and serial number *S*_NO_. After recording the data, the administrator uploads it to the cloud, which produces the *K*_*M*_ and unique identifiers for the doctor (*DR*_*I*  *D*_), patient (*PT*_*I*  *D*_), and ward boy (*NS*_*I*  *D*_) and sends them to the admin. KCF is used by the administrator to generate several subkeys (*K*_*S*_) for the secure communication between the gateway and other organizations. Users (patient, doctor, etc.) receive identification details and unique secret subkeys from the administrator, while the gateway gets the *K*_*M*_, *K*_*S*_, *DR*_*I*  *D*_, *PT*_*I*  *D*_, *NS*_*I*  *D*_, and *HP*_*I*  *D*_. The unique IDs assist the administrator in ensuring the privacy of the patient's records during the offline registration phase. Only those ward boys and doctors treating that patient are given access to the patient by the administrator. The suggested approach allows the administrator to pick which stakeholders can access the cloud-based information.  Table 4 shows the administrator's default settings, which include granting access and storage privileges to doctors treating the patient. On the other hand, other stakeholders have merely been provided access to the information.

The article "On the Design of Secured and Reliable Dynamic Access Control Scheme of Patient E-Healthcare Records in Cloud Environment" was retracted in 2023. Reasons: signs of a paper mill; suspected computer-generated content; unreliable results or conclusions; concerns about the data.

### 4.3. Data Retrieval Phase

It is shown in Figure 5 that the doctor visits the gateway to express interest in communicating with a cloud-based service. The nonce *N*_CC1_ is generated by the doctor's device, and it is concatenated with *DR*_*I*  *D*_ and *PT*_*I*  *D*_ to compute *γ*. For computing Γ, the resulting message *γ* is encrypted (*K*_*S*_, *γ*). *H*_*S*_ (*DR*_*I*  *D*_) has been calculated and saved in O using the hash function. Γ is combined with the message O for producing A. The gateway receives the message *S*1 from the user, which contains the value A. The gateway retrieves *DR*_*I*  *D*_ from the database, calculates its hash value, and saves it in *Z*. To determine the right subkey for decryption, the gateway compares Z with O (*Z* = = *O*) using the subkey *K*_*S*_, to form *δ*, and Γ is decrypted. The gateway examines the nonce *N*_CC1_ for freshness; if it is fresh, then the procedure is restarted; otherwise, it is aborted. The nonce *N*_CC2_ is generated by the gateway and is concatenated with some other values *HP*_*I*  *D*_‖*DR*_*I*  *D*_‖*PT*_*I*  *D*_‖*N*_CC2_ and form *ζ*. Subsequently, *M*_*K*_ is used for the encryption of *ζ* in order to form *η*. The gateway has now sent message *S*2 to the cloud. Cloud decrypts the message *η* using *M*_*K*_ after receiving it to give *ϑ*. The procedure is continued if *N*_CC2_ is fresh; otherwise, it is aborted. The variables *HP*_*I*  *D*_, *PT*_*I*  *D*_, and *DR*_*I*  *D*_ are checked, and if they are determined to be false, the procedure is aborted. It is checked to see whether *PT*_*I*  *D*_ belongs to *DR*_*I*  *D*_, and if it does, the procedure is continued. Nonce (*N*_CC3_) and requested data (*D*_*R*_) are generated after successful verification and are concatenated with other values *HP*_*I*  *D*_‖*PT*_*I*  *D*_‖*DR*_*I*  *D*_‖*D*_*R*_‖*N*_*CC*3_ to form Θ. To generate *κ*, the Θ calculated is encrypted with *M*_*K*_. The gateway receives message *S*3 from the cloud. When gateway receives a message, it decrypts it using *D*_YP_(*K*_*M*_, *κ*) to form *μ*. When *N*_CC3_ is checked, if it is found to be fresh, the operation is continued; otherwise, it is paused. The gateway now verifies *HP*_*I*  *D*_ and generates *N*_CC4_ as a nonce. Subsequently, ∅ is calculated by concatenating all of the values *DR*_*I*  *D*_‖*PT*_*I*  *D*_‖*D*_*RQ*_‖*N*_*CC*4_, and then, ∅ is encrypted using *K*_*S*_ to form ∅. The doctor receives the message *S*4 from the gateway and decrypts the message ∅ using *K*_*S*_ and computes *ρ*. Only if nonce *N*_CC4_ is still alive, the operation is continued further. The doctor can successfully retrieve the requested data, *D*_RQ_, after verifying the freshness.

The article "On the Design of Secured and Reliable Dynamic Access Control Scheme of Patient E-Healthcare Records in Cloud Environment" was retracted in 2023. Reasons: signs of a paper mill; suspected computer-generated content; unreliable results or conclusions; concerns about the data.

### 4.4. Data Storage Phase

It is shown in Figure 5 that the doctor visits the gateway to engage in communicating with a cloud-based service. The nonce *N*_CC1_ is generated by the doctor's device, and it is concatenated with *DR*_*I*  *D*_ and *PT*_*I*  *D*_ to compute *γ*. For computing Γ, the message resulting *γ* is then encrypted (*K*_*S*_, *γ*). *H*_*S*_(*DR*_*I*  *D*_) has been calculated and saved in *O* using the hash function. Γ is merged with the message *O* to produce *A*. The gateway receives message *S*1 from the user, which contains the value *A*. The gateway extracts *DR*_*I*  *D*_ through the database for calculating and storing its hash value in *Z*. To determine the right subkey for decryption, the gateway compares *Z* with O (*Z* == O). The gateway examines the nonce *N*_CC1_ for freshness; if it is fresh, the procedure is restarted; otherwise, it is aborted. The nonce *N*_CC2_ is generated by the gateway and is concatenated with some other values *HP*_*I*  *D*_‖*DR*_*I*  *D*_‖*PT*_*I*  *D*_‖*N*_CC2_ and form *ζ*. Subsequently, *M*_*K*_ has been used to encrypt *ζ* for formation of *η*. The message *S*2 is now sent to the cloud by the gateway. Cloud decrypts the message *η* using *M*_*K*_ after receiving it to give *ϑ*. The procedure is continued if *N*_CC2_ is fresh; otherwise, it is aborted. The variables *HP*_*I*  *D*_, *PT*_*I*  *D*_, and *DR*_*I*  *D*_ are checked, and if they are determined to be false, the procedure is aborted. It is checked to see whether *PT*_*I*  *D*_ belongs to *DR*_*I*  *D*_, and if it does, the procedure is continued. Nonce (*N*_CC3_) and requested data (*D*_*R*_) are generated after successful verification and are concatenated with other values *HP*_*I*  *D*_‖*PT*_*I*  *D*_‖*DR*_*I*  *D*_‖*D*_*R*_‖*N*_CC3_ to form Θ. To generate *κ*, the Θ calculated is encrypted with *M*_*K*_. The gateway receives message S3 from the cloud. When gateway receives a message, it decrypts it using *D*_*YP*_(*K*_*M*_, *κ*) to form *μ*. When *N*_CC3_ is checked, if it is found to be fresh, the operation is continued; otherwise, it is paused. The gateway now verifies *HP*_*I*  *D*_ and generates *N*_CC4_ as a nonce. Subsequently, ∅ is calculated by concatenating all of the values *DR*_*I*  *D*_‖*PT*_*I*  *D*_‖*D*_*RQ*_‖*N*_*CC*4_, and then, ∅ is encrypted using *K*_*S*_ to form ∅. The doctor receives the message S4 from the gateway after that. The doctor decrypts message ∅ using *K*_*S*_ and computes *ρ*. Only if nonce *N*_*CC*4_ is still alive, the operation is continued further. After verifying the freshness, the doctor can successfully retrieve the requested data, *D*_RQ_.

The article "On the Design of Secured and Reliable Dynamic Access Control Scheme of Patient E-Healthcare Records in Cloud Environment" was retracted in 2023. Reasons: signs of a paper mill; suspected computer-generated content; unreliable results or conclusions; concerns about the data.

## 5. Experimental Setup

We have developed a cloud-based web application hosted on third-party AWS cloud infrastructure. Web application is developed using PHP version 7.3. The main aim of this web application is to store and protect the e-healthcare records of the patient over a third-party cloud. The web application uses a dynamic access control scheme for sharing and uploading e-healthcare data over the cloud. Our web application service was hosted and tested on Elastic Compute Cloud (EC2) instances provided on Amazon Web Services (AWS). On the cloud platform, the virtual environment is provided by an instance of Amazon's Elastic Compute Cloud (EC2). We used EC2 instances to conduct experiments in our experimental evaluation, as shown in Table 5.

## 6. Experimental Design

We ran three sets of experiments to assess the web application's performance. When we conduct an experiment, we use a preallocated Amazon EC2 instance to run an artificial workload to measure the throughput (requests per second) and average web application response time. For artificial workload generation, we have used [63] for web application service performance measurement. It is possible to create an artificial user session to mimic the process of searching for an existing patient and adding a new patient record to the system. It is possible to simultaneously add a new patient to the system while conducting a patient search that returns a significant number of results from the database. The details of all the three experiments are described in Table 6.

### 6.1. Experiment 1: An EC2 Medium Instance with a Predetermined Allocation

As part of experiment 1, EC2 instances assigned to the web and database tiers are shown in the following Figures 6–8 which show throughput with average response time and CPU use for the EC2 instances. The figure shows that by the 15^th^ minute of the study, the throughput has stopped rising linearly, significantly increasing the application's response time. An obvious constraint has been discovered in the web server tiers that CPU use approaches 100%, indicating a bottleneck. After 29^th^ minutes, the web server tier instance has stopped responding, and we cannot receive throughput and response time measures after that point in time. Howsoever, we can still monitor both instances of CPU consumption with the Amazon CloudWatch. This experiment achieved a maximum throughput of 934 requests per second.

The article "On the Design of Secured and Reliable Dynamic Access Control Scheme of Patient E-Healthcare Records in Cloud Environment" was retracted in 2023. Reasons: signs of a paper mill; suspected computer-generated content; unreliable results or conclusions; concerns about the data.

### 6.2. Experiment 2: An EC2 Large Instance with a Predetermined Allocation

Figures 9–11 illustrate throughput, average response time, and CPU consumption for EC2 instances assigned to the web and database tiers in Experiment 2. The throughput stops increasing linearly by the 21^th^ minute of the experiment, and there was no significant increase in response time throughout this experiment. As of this writing, the typical response time remains under around 45 milliseconds. There has been no discernible increase in CPU use in the web server with database tier replicas. This experiment gained a maximum throughput of 1051 requests per/second. Because bandwidth became a big issue at the 21^th^ minute of the experiment and the web server instance is using 245 MB/seconds and 486 MB/second on an average for network input and output, ideally throughput should have continued to rise throughout the experiment.

### 6.3. Experiment 3: An EC2 xlarge Instance with a Predetermined Allocation

Data from Experiment 3's EC2 instances are shown in Figure 12 for the throughput, average response time, and CPU utilization of the web and database tiers of EC2 instances, respectively, as depicted in Figures 13 and 14. In this experiment, there is no hint of a significant rise in response time at the point where throughput stops rising linearly at 21^th^ minute. As of this writing, the typical response time is around 45 milliseconds. A lack of CPU saturation has been found within web and database tiers of the application. In this experiment, we achieved a maximum throughput of 1150 requests/per second. Because we see the identical bandwidth constraint in this experiment as we did in Experiment 2, the results are very similar. The conclusion is clear: increasing the web tier instance's resources does nothing to alleviate bandwidth constraints.

### 6.4. Comparing Cloud-Based Web Application with Blockchain Platform

EHR and EMR interoperability and security issues have been addressed by blockchain technology, which has seen tremendous growth in the healthcare industry. Before blockchain can realize its full potential and be used in medical care, it must overcome various barriers. In this section, in terms of latency, throughput, and execution time, we test and compare the performance of the blockchain platform and web application hosted on the third-party cloud platform AWS using a secure scheme implemented for patient health records in the cloud environment. To evaluate our cloud-based web application with the Ethereum blockchain platform, we compared execution time, throughput, and latency of paper [64]. Paper [64] deployed Ethereum smart contracts using IoT devices. The purpose of paper [64] is to evaluate, store, and access transactions. We compare our patient's records, which are stored and accessed from a third-party cloud with paper [64]. The main focuses for comparing cloud-based web application with Ethereum blockchain platform are as follows:

1. Ethereum and cloud-based web application comparison analysis.
2. Performance matrices based on latency, throughput, and execution time are used to analyze the number of user transactions.

The article "On the Design of Secured and Reliable Dynamic Access Control Scheme of Patient E-Healthcare Records in Cloud Environment" was retracted in 2023. Reasons: signs of a paper mill; suspected computer-generated content; unreliable results or conclusions; concerns about the data.

JMeter tools are being used in an experiment to protect patient e-health records hosted on third-party cloud providers' AWS. We then examined paper [64] Ethereum performance. We assessed latency, execution time, and throughput by different loads, such as the number of queries fired by the user on Amazon AWS cloud, for the performance evolution of cloud and blockchain technologies. The system configuration is shown in Table 7 for comparing blockchain platforms and third-party cloud platform AWS. For comparing the cloud-based web application system, we store and access e-health records of a patient analyzed with store and access transaction of Ethereum blockchain platform using IoT devices. Figures 15–19 show analysis Figures 20 of latency, execution time, and throughput of store and access transaction of third-party cloud AWS and Ethereum with IoT devices. We can see as per Figures 15 and 16 the latency of access and store transaction comparison. As the dataset rises in size, so does the latency of both platforms, which can be seen in the graph. As transaction gets increases latency performance of the third-party cloud-based platform is less compared to the Ethereum blockchain platform, increasing the number of transactions prompts us to look into the impact on transaction execution time variances that might exist. On both systems, as the number of transactions in the dataset grows, Figures 17 and 18 execution times are longer. Finally, the number of completed transactions per second, starting with the first deployment time, is used to determine throughput. Here, in Figures 19 and 20, it is shown that when the number of transactions is varied, the throughput remains relatively constant as the number of transactions increases; the throughput of access transactions is greater than that of store transactions in both the platforms. As transaction increases, the throughput performance of a third-party cloud-based platform is greater compared to the Ethereum blockchain platform. Secured and reliable dynamic access control scheme of patient e-healthcare records implemented in third-party cloud-based e-health application performs better in cloud environment compared to Ethereum blockchain platform using IoT devices. Finally, based on JMeter tool results, we can deduce that a cloud-based web application hosted on AWS for secure sharing of patient health records over a third-party cloud platform has the edge over the Ethereum blockchain platform.

The article "On the Design of Secured and Reliable Dynamic Access Control Scheme of Patient E-Healthcare Records in Cloud Environment" was retracted in 2023. Reasons: signs of a paper mill; suspected computer-generated content; unreliable results or conclusions; concerns about the data.

## 7. Conclusions

To demonstrate the performance of our web application service, we used Amazon EC2 instances of various sizes to simulate growing workloads. We believe this study will assist web application service providers in utilizing proper cloud resources to provide response time guarantees while minimizing operational costs. Patient medical records can be easily accessed from anywhere with cloud-based e-healthcare services. Since cloud service providers offer cost-effective solutions, cloud-based e-health care has become possible. Despite the many benefits, the cloud storage and retrieval framework are particularly sensitive to wireless channels. Patient data can only be stored and accessed by those who have been granted permission (such as the patient, ward boys, doctors, and close family members). The hospital's responsibility for keeping records of patients is reduced, and access to storage of health records is improved. The proposed scheme's reliability against numerous significant attacks such as message alteration, MITMA, and replay, among others, was revealed by security analysis. The method has enormous potential for cloud-based solutions. The proposed secure access methodology for storing and accessing patient's e-health records over third-party clouds is compared to the performance evaluation of two natural traffic flow, store, and access transactions proposed using the Ethereum blockchain platform with IoT device. It can be seen that, despite having a standard system configuration, the cloud platform performs significantly better than Ethereum in relation to execution time, throughput, and latency. Eventually, in future work, we want to test newer versions of Hyperledger Fabric with a cloud-based solution and look into different scenarios like how having numerous functions in the network affects the network's overall performance of both platforms. Furthermore, we want to compare the performance of cloud-based e-health solutions for the patient with different public blockchain technology for a higher number of transactions. Other analyses related to data security and privacy are on our agenda for the near future, particularly in the context of external access to e-healthcare data transferred through various networks over the cloud.

The article "On the Design of Secured and Reliable Dynamic Access Control Scheme of Patient E-Healthcare Records in Cloud Environment" was retracted in 2023. Reasons: signs of a paper mill; suspected computer-generated content; unreliable results or conclusions; concerns about the data.

## Figures and Tables

**Figure 1:** Cloud-based electronic health data architecture.

**Figure 2:** E-healthcare system based on the cloud for secure sharing with different entities.

**Figure 3:** Registration for hospital over cloud.

**Figure 4:** Device registration (offline).

**Figure 5:** Retrieval phase for data.

**Figure 6:** Throughput (requests per second).

**Figure 7:** Avg. response time.

**Figure 8:** Web server and database tier instances' CPU utilization.

**Figure 9:** Throughput (requests per second).

**Figure 10:** Avg. response time.

**Figure 11:** Web server and database tier instances' CPU utilization.

**Figure 12:** Throughput (requests per second).

**Figure 13:** Avg. response time.

**Figure 14:** Web server and database tier instances' CPU utilization.

**Figure 15:** Latency comparison of access transaction.

**Figure 16:** Latency comparison of store transaction.

**Figure 17:** Execute time comparison of access transaction.

**Figure 18:** Execute time comparison of store transaction.

**Figure 19:** Throughput comparison of access transaction.

**Figure 20:** Throughput comparison of store transaction.

**Table 1:** Analyzing protocols based on security features.

Scheme	*J*_1_	*J*_2_	*J*_3_	*J*_4_	*J*_5_
*J*_*S*_	Yes	Yes	*R*	Yes	Yes
[12]	No	No	*R*	No	No
[47]	No	Yes	*W*_*O*_	No	Yes
[14]	No	Yes	*R*	Yes	Yes
[48]	No	Yes	*W*_*O*_	No	Yes
[49]	No	Yes	*R*	Yes	Yes
[50]	No	Yes	*R*	Yes	Yes
[28]	No	Yes	*W*_*O*_	Yes	No
[50]	No	Yes	*W*_*O*_	No	No
[51]	No	Yes	*W*_*O*_	Yes	Yes
[52]	No	Yes	*W*_*O*_	Yes	Yes
[53]	No	Yes	*W*_*O*_	Yes	Yes

Abbreviations: *J*_1_: secrecy, *J*_2_: integrity, *J*_3_: authentication, *J*_4_: confidentiality, *J*_5_: authorization, *J*_*S*_: proposed scheme, Yes: complying to the properties of security, No: non-complying to the properties of security, *R*: mutual, *W*_*O*_: one way.

**Table 2:** Evaluation of related study.

Framework	E-healthcare	Security risks	Awareness	Challenges	Impacts
[54]	R	ii	G	F	E
[55]	R	i	G	E	E
[56]	R	vii	F	E	G
[57]	P	ii	G	F	G
[58]	R	vi	F	E	F
[59]	I	iii	G	E	E
[60]	C	v	E	E	G
[61]	M	iv	G	F	E
[62]	M	i	G	E	F

Abbreviations: R: RFID, P: pacemaker, I: IP, M: embed medical devices, C: embed cardiac defibrillators, i: identification issues, ii: radio frequency attack, iii: intercepting attack, iv: device duplication issue, v: electromagnetic interruption, vi: illegal remote surveillance, E: high, F: medium, G: lower.

**Table 3:** Description of annotations.

Annotations	Description
‖	Concatenation operation
KY_GT_	Temporary key of gateway
KY_AT_	Temporary key of administration
*H*_*S*_	Hash
*S*_NO_	Serial number
*D*_*S*_	Data to be stored
RR_*N*_	Reference receipt number
RP_*N*_	Payment receipt number
*D*_YP_	Decryption
*E*_YP_	Encryption
*N*_CC_	Nonce
CK_PU_	Public key of cloud
CK_PR_	Private key of cloud
ID_UG_	Unique ID issued by government
ID_UH_	Unique ID issued by hospital
*K*_*M*_	Master key
*K*_*S*_	Subkey
*D*_FK_	Key derivation function
*D*_RQ_	Requested data
DR_ID_	Doctor ID
PT_ID_	Patient ID
HP_ID_	Hospital ID

The article "On the Design of Secured and Reliable Dynamic Access Control Scheme of Patient E-Healthcare Records in Cloud Environment" was retracted in 2023. Reasons: signs of a paper mill; suspected computer-generated content; unreliable results or conclusions; concerns about the data.

**Table 4:** Access rights distribution.

Device	Read	Write
Patient	Yes	No
Doctor	Yes	Yes
Ward boy	Yes	No

**Table 5:** Resource allocation and cost.

Type of instances	vCPU (core)	RAM	Storage	Cost in (USD/hour)
m3.medium	1	3.12	4	0.071
m3.large	2	7.35	32	0.137
m3.xlarge	4	16	600	0.476

**Table 6:** Details on the experiment.

Number	Experiment	Description
1	Using the EC2 medium instance for a fixed amount of storage	Preallocated EC2 instances of type m3.medium and m3.2xlarge are preallocated in the web service layer and the database layer, respectively
2	Statically allocating resources with an Amazon EC2 large instance	We have preallocated two EC2 instances, one for web services and the other for databases, both of which are of type m3.2xlarge
3	EC2 xlarge instance for static allocation	Preallocated EC2 instances of type m3.2xlarge for the database and one of type m3.2xlarge for the web service tier

**Table 7:** System configuration.

Parameter	AWS	Ethereum 1.8.3
RAM	16 GB	16 GB
OS	Ubuntu Linux	Raspberry PI 3
Virtual CPU	4	8
Apache2	2.4.38	2.4.52
Storage	600 GB	1 TB

## Data Availability

No data were used to support the findings of the study.
